The article "Restoration Algorithm-Based Ultrasound Image in Evaluating the Effect of Dexmedetomidine on Patients with Neurological Disorder Anesthetized by Sevoflurane" was retracted in 2023. Reasons: signs of a paper mill; compromised peer review; unreliable results or conclusions.

# Restoration Algorithm-Based Ultrasound Image in Evaluating the Effect of Dexmedetomidine on Patients with Neurological Disorder Anesthetized by Sevoflurane

**DOI:** 10.1155/2022/1320893

**Published:** 2022-02-21

**Authors:** Yingying Yao, Zhihui Sun, Yanming Huang, Xiaoqin Zhou, Daolin Xia

**Affiliations:** ^1^Department of Anesthesiology, The First People's Hospital of Xuzhou, Xuzhou, 221000 Jiangsu, China; ^2^Department of Anesthesiology, People's Hospital of Xuyi County, Xuyi, 211700 Jiangsu, China

## Abstract

The study focused on the application value of ultrasound images processed by restoration algorithm in evaluating the effect of dexmedetomidine in preventing neurological disorder in patients undergoing sevoflurane anesthesia. 90 patients undergoing tonsillectomy anesthesia were randomly divided into normal saline group, propofol group, and dexmedetomidine group. The ultrasound images were processed by restoration algorithm, and during the postoperative recovery period, ultrasound images were used to evaluate. The results showed that the original ultrasonic image was fuzzy and contained interference noise, and that the image optimized by restoration algorithm was clear, without excess noise, and the image quality was significantly improved. In the dexmedetomidine group, the extubation time was 10.6 ± 2.3 minutes, the recovery time was 8.4 ± 2.2 minutes, the average pain score during the recovery period was 2.6 ± 0.7, and the average agitation score was 7.2 ± 2.4. Of 30 patients, there were 13 cases with vertigo and 1 case with nausea and vomiting. The vascular ultrasound imaging showed that, in the dexmedetomidine group, the peak systolic velocities (PSV) of the bilateral vertebral arteries during the recovery period were 67.7 ± 14.3 and 67.9 ± 15.2 cm/s, respectively; the end-diastolic velocities (EDV) of the bilateral vertebral arteries were 27.8 ± 6.7 and 24.69 ± 5.9 cm/s, respectively; the PSV in bilateral internal carotid artery systolic peak velocities were 67.2 ± 13.9 and 67.8 ± 12.7 cm/s, respectively; the EDV in bilateral internal carotid arteries were 27.7 ± 5.3 and 26.9 ± 4.9 cm/s, respectively; bilateral vertebral artery resistance indexes (RIs) were 0.6 ± 0.02 and 0.71 ± 0.08, respectively; the bilateral internal carotid artery RIs were 0.57 ± 0.04 and 0.58 ± 0.06, respectively, all better than the normal saline group (12.1 ± 2.5 minutes, 10.1 ± 2.3 minutes, 3.9 ± 0.6, 10.6 ± 3.7, 15 cases, 11 cases, 81.5 ± 13.6, 80.7 ± 11.6 cm/s, 29.3 ± 6.8, 28.9 ± 6.7 cm/s, 74.3 ± 10.2, 73.9 ± 12.5 cm/s, 29.1 ± 4.3, 29 ± 4.5 cm/s, 0.84 ± 0.06, 0.83 ± 0.05, 0.8 ± 0.04, and 0.81 ± 0.05) and the propofol group (11.4 ± 2.1 minutes, 9.0 ± 2.1 minutes, 3.4 ± 0.8, 8.5 ± 2.3, 12 cases, 9 cases, 72.5 ± 12.9, 73.4 ± 11.8 cm/s, 28.6 ± 5.4, 26.5 ± 5.1 cm/s, 72.1 ± 11.4, 73.5 ± 10.6 cm/s, 28.8 ± 5.6, 27.3 ± 4.7 cm/s, 0.78 ± 0.07, 0.82 ± 0.06, 0.76 ± 0.03, and 0.78 ± 0.05), and the differences were statistically significant (*P* < 0.05). In conclusion, ultrasound images processed by restoration algorithm have high image quality and high resolution. The dexmedetomidine can prevent neurological disorder in patients with sevoflurane anesthesia and is suggested in postoperative rehabilitation.

The article "Restoration Algorithm-Based Ultrasound Image in Evaluating the Effect of Dexmedetomidine on Patients with Neurological Disorder Anesthetized by Sevoflurane" was retracted in 2023. Reasons: signs of a paper mill; compromised peer review; unreliable results or conclusions.

## 1. Introduction

Sevoflurane is an inhaled anesthetic, which is widely used in clinical anesthesia. It is colorless, transparent, and aromatic, and therefore, it is easy to be accepted by patients. It has a low blood partition coefficient, causing small irritation to the airway, and it can relax the airway smooth muscle. Additionally, it induces anesthesia quickly and the patient will recover consciousness in short time. Hence, it is suitable for surgery [1, 2]. However, such nontracheal general anesthesia drugs also have disadvantages; that is, there may be transient neurological disorder during the postoperative recovery period [3, 4]. Clinically, neurological disorder manifests as vertigo, headache, palpitation, instable hemodynamics, agitation, and gastrointestinal dysfunction, such as nausea and vomiting [5]. Studies have shown that the use of sevoflurane will increase the excitability of the sympathetic nervous system in patients, which in turn leads to neurological disorder [6]. Discomfort of patients during the postoperative recovery period was often considered normal. Nevertheless, with the advancement of medical technology, there are higher requirements for comfort and safety of patients, and thus, clinical anesthesia becomes a focus.

Dexmedetomidine is an *α*2 adrenergic receptor agonist. It has good sedative and analgesic effects. Compared with other similar drugs, it exhibits higher selectivity. For patients undergoing general anesthesia, it is used to sedate during tracheal intubation and mechanical ventilation. It has high application value in clinical anesthesia [7, 8]. As for neurological disorder that occurs in patients after surgery, clinically, imaging methods, such as cervical vascular ultrasound, are usually used to determine the severity of neurological disorder factoring into hemodynamics. Ultrasound has an important application value in clinical surgery. It can extract a wide range of information and is simple to operate, with no damage to patients and low cost. It is used to guide the formulation of surgical plan and improve surgical efficacy. However, due to problems such as the aging of imaging equipment or components, the quality of the ultrasound image is always unsatisfactory. There are problems of low resolution and interference noise, resulting in deviations in the information and data obtained, while the emergence of restoration algorithm solves these problems. Because the point spread function of the degradation factor that causes low image quality has a certain degree of similarity at a certain depth, it regards all point spread functions as a whole. Through image-block iterations, a clear ultrasound image after restoration is obtained [9–11]. Incorporating this algorithm into ultrasound imaging technology can reduce interference noise, enhance the resolution, and improve the accuracy of detection.

The article "Restoration Algorithm-Based Ultrasound Image in Evaluating the Effect of Dexmedetomidine on Patients with Neurological Disorder Anesthetized by Sevoflurane" was retracted in 2023. Reasons: signs of a paper mill; compromised peer review; unreliable results or conclusions.

In this experiment, the restoration algorithm was used to process the ultrasound images of 90 patients undergoing tonsillectomy. The subjects were randomly divided into three groups, namely, the normal saline group, the propofol group, and the dexmedetomidine group. Indicators during the recovery period were compared, to verify the effects of dexmedetomidine in the recovery of neurological disorder in patients with sevoflurane anesthesia. This study provides a reference for the investigation of the sedative and analgesic effects of dexmedetomidine.

## 2. Materials and Methods

### 2.1. Research Subjects

Ninety patients undergoing tonsillectomy in the hospital from June 2018 to December 2020 were selected as research subjects and randomly divided into three groups, with each 30 (the normal saline group: sevoflurane plus intraoperative normal saline, the control group: sevoflurane plus propofol, and the experimental group: sevoflurane plus dexmedetomidine). During the postoperative recovery period, ultrasound images processed by restoration algorithm were used for evaluation. The subjects were selected as per the following inclusion criteria: (i) patients aged 18-70 years, (ii) patients of American Medical Association Anesthesia Classification I-II, (iii) patients free of symptoms such as cold and fever within one week before surgery, (iv) patients with normal routine examination results on admission, (v) patients without other organic diseases, and (vi) patients with complete clinical data. The exclusion criteria are as follows: (i) patients combined with other serious organic diseases, (ii) patients with a history of allergy to relevant drugs, (iii) patients of American Medical Association Anesthesia Classification ≥ III, (iv) patients with symptoms such as cold and fever before surgery, (v) patients not willing to cooperate and with poor compliance, and (vi) patients with incomplete clinical data. The patients and their family members had been informed of all details of the study and signed the informed consent form. This study was approved by the ethics committee of the hospital.

The article "Restoration Algorithm-Based Ultrasound Image in Evaluating the Effect of Dexmedetomidine on Patients with Neurological Disorder Anesthetized by Sevoflurane" was retracted in 2023. Reasons: signs of a paper mill; compromised peer review; unreliable results or conclusions.

### 2.2. Methods of Anesthesia

All subjects were forbidden to eat 8 hours before surgery and to drink 4 hours before surgery. First, 5% glucose injection was intravenously injected, and vital signs were recorded, such as heart rate, electrocardiogram, blood oxygen saturation, and blood pressure. The patient inhaled 2-3% sevoflurane through a face mask, with the oxygen flow set to 7 L/min, and 2 *μ*g/kg of fentanyl was intravenously injected at the same time. In the experimental group, 0.3 *μ*g/kg dexmedetomidine was intravenously injected, the eyelash reflex and swallowing reflex disappeared, and 0.1 mg/kg cisatracurium was administered. Subsequently, the tracheal intubation was performed and the ventilator was used for mechanical ventilation. During the operation, 3% sevoflurane was used to maintain anesthesia, and the vital signs of the patient should be kept stable. In the control group, ten minutes before the end of the operation, 0.25 mg/kg propofol was intravenously injected. After the operation, the inhalation of sevoflurane was stopped and the patient was sent to the anesthesia care unit. The tracheal tube can be removed after the patient's voluntary consciousness, swallowing reflex, and muscle strength gradually recovered.

### 2.3. Data Collection

The operation time, extubation time, and the recovery time from stop inhaling sevoflurane to opening the eyes were recorded. The number of cases with pain, agitation, vertigo, and nausea and vomiting was counted. The scoring criteria for pain are as follows: the lowest score was 0, which means there is no pain; the highest score was 10, which means the pain was severe and unbearable. The scoring criteria for agitation are shown in Table 1.

### 2.4. Ultrasound Examination of the Blood Vessels

Doppler ultrasound system was used, and the frequency of the linear array probe was 3-12 MHz. After the patient was fully calm for 5 minutes, he lied on his back, and his jaw was lifted to fully expose the neck. An experienced imaging doctor used a linear array probe to measure the peak systolic velocity (PSV), end-diastolic velocity (EDV), and resistance index (RI) of the bilateral vertebral arteries and bilateral internal carotid arteries of all patients. The measurement was repeated three times, and the average was taken.

### 2.5. Restoration Algorithm

During ultrasound imaging, aging or failure of components, signal movement between the imaging object and the image sensor, and interference noise can all degrade the quality of ultrasound images. The factor that degrades the quality of ultrasound images is called the point spread function. Any image degradation factor has its point spread function mode. Here, all the point spread function modes are regarded as a whole system, and the system model is expressed as follows.

(1) $$\begin{array}{c} A\left(x,y\right)=\iint_{-\infty }^{\infty }B\left(x,y\right)C\left(x,y\right)e_{x}e_{y}+D\left(x,y\right), \end{array}$$

where *A*(*x*, *y*) is a low-quality ultrasound image, *B*(*x*, *y*) is a clear ultrasound image, *C*(*x*, *y*) is a point spread function, *D*(*x*, *y*) is a redundant interference noise, and ⊗ is a convolution method. The equation can be simplified as follows.

(2) $$\begin{array}{c} A=B⊗C+D. \end{array}$$

The restoration algorithm is the reverse operation of the above equation, called deconvolution, during which an optimal criterion is regarded as a constraint on the low-quality ultrasound image to derive a clear image before degradation. In the process of deconvolution, the blind solution method is commonly used, where only the low-quality image is known, and the point spread function mode and the clear ultrasound image are unknown. For such ill-posed problems, regularization methods are generally used. It is to derive a solution of an adaptive problem similar to the ill-posed problem, and then, this solution is used to deduce the solution of the ill-posed problem. Finally, the restoration algorithm model to obtain the clear ultrasonic image is expressed as follows.

(3) $$\begin{array}{c} \underset{B,C}{\arg\min}{\left\|A⊗C-B\right\|}_{2}^{2}, \end{array}$$

where ‖•‖_2_ is the norm of the matrix. In practice, when dealing with low-quality ultrasound images, it is usually necessary to import corresponding experience and historical data, so that the clear images after restoration can be acquired efficiently. At this time, a regularization method is required. The derivation model of the regularization method in the restoration algorithm is as follows:

(4) $$\begin{array}{c} \underset{B,C}{\min}\left\{{\left\|A-B⊗C\right\|}_{2}^{2}+\lambda {\left\|TB\right\|}^{2}\right\}, \end{array}$$

where *λ* is the parameter of regularization and *T* is the matrix of regularization. In the selection of regularization parameters, experience and historical data are usually used, and regular weights are set within the delineated value range. The optimal result is selected as the parameter according to the clarity of the restored image. The quality of the ultrasound image is evaluated based on the difference between the reference image and the restored image. Generally, the peak signal-to-noise ratio (PSNR) is a commonly used indicator. It is simply defined by mean square error (MSE), expressed as follows.

(5) $$\begin{array}{c} \text{PSNR}=10\cdot \log_{10}\left(\frac{{{\mathrm{MAX}}_{B}}^{2}}{{\text{MSE}}_{B}}\right), \end{array}$$

where MAX_*B*_ is the highest pixel value of the ultrasound image and MSE_*B*_ is the mean square error between the restored image and the reference image, which can be expressed as follows.

(6) $$\begin{array}{c} {\text{MSE}}_{B}=\frac{1}{fg}\overset{f-1}{\underset{h=0}{\sum }}\overset{l=g-1}{\underset{l=0}{\sum }}{\left\|B\left(h,l\right)-B\left(h,l\right)\right\|}^{2}, \end{array}$$

where (*f*, *g*) is the size of the image. A higher PSNR value indicates higher quality of the ultrasound image after restoration. A lower MSE value indicates smaller differences and higher similarity between the two. In the study, the MSE is used to evaluate the accuracy of the point spread function, which is expressed as follows.

(7) $$\begin{array}{c} {\text{MSE}}_{C}=\frac{1}{F*G}\overset{F}{\underset{h=1}{\sum }}\overset{G}{\underset{l=1}{\sum }}{\left(C\left(h,l\right)-C\left(h,l\right)\right)}^{2}. \end{array}$$

However, if the displayed image is distorted due to some unavoidable problems of the ultrasound equipment during imaging, the reference evaluation standard cannot be used. Therefore, the resolution gain (RG) is used to evaluate the quality of the restored ultrasound image. It is defined as the ratio between the total numbers of pixels with an autocorrelation value greater than 0.75 in the original image signal to the deconvoluted signal. A higher RG value indicates higher quality of the ultrasound image after restoration. The expression is as follows:

(8) $$\begin{array}{c} \text{RG}=\frac{\text{Total}\left(\text{autocorrelation}\left(A\right)>0.75\right)}{\text{Total}\left(\text{autocorrelation}\left(B\right)>0.75\right)}, \end{array}$$

where autocorrelation(*A*) represents the autocorrelation value of matrix *A* and total(*A*) is the total number of all factors in matrix *A*. Providing that there is a linear degradation model of ultrasound images, expressed as Equation (2), the image experience and historical data in Equation (3) can be used to constrain to construct a restoration regularization model, expressed as follows:

(9) $$\begin{array}{c} \underset{B,C}{\arg\min}\lambda {\left\|B⊗C-A\right\|}_{2}^{2}+\frac{{\left\|B\right\|}_{1}}{{\left\|B\right\|}_{2}}+\theta {\left\|C\right\|}_{1}, \end{array}$$

where argmin is the least squares format of the model and the second term is the constraint term for high-quality ultrasound images. Generally, when dealing with such a nonconvex problem, *B* and *C* must be initialized first and then optimized and upgraded. The derivation of *B* and *C* is usually called the *B* subproblem and the *C* subproblem. When deriving *B*, the point spread function *C* is regarded as known, and the derivation equation is expressed as follows:

(10) $$\begin{array}{c} \underset{B}{\arg\min}\lambda {\left\|B⊗C-A\right\|}_{2}^{2}+\frac{{\left\|B\right\|}_{1}}{{\left\|B\right\|}_{2}}. \end{array}$$

When dealing with such regularization problems, iterative shrinkage-thresholding algorithm (ISTA) is often used, which is an algorithm with high computational efficiency. Equation below is obtained by setting ‖*B*‖_2_ as the value after the last iteration.

(11) $$\begin{array}{c} \underset{B}{\arg\min}\lambda {\left\|B⊗C-A\right\|}_{2}^{2}+{\left\|B\right\|}_{1}. \end{array}$$

Equation (11) optimized by ISTA is expressed as follows.

(12) $$\begin{array}{c} B^{n+1}=J_{\alpha jl}\left(A-{jc}^{J}\left({CB}^{n}-A\right)\right), \end{array}$$

where *J*_*αjl*_ is the contraction factor, expressed as follows.

(13) $$\begin{array}{c} J_{\alpha }\left(x\right)l=\max\left(\left|x_{l}\right|-x,0\right)\mathrm{sign}\left(x_{l}\right). \end{array}$$

In short, the iterative shrinkage threshold algorithm can be used as the internal iteration of the *B* algorithm when deriving *B*. After *B* is optimized, the point spread function *C* can be optimized. So, the loss function of the *C* subproblem is expressed as follows.

(14) $$\begin{array}{c} \underset{C}{\arg\min}\lambda {\left\|B⊗C-A\right\|}_{2}^{2}+\theta {\left\|C\right\|}_{1}. \end{array}$$

In this derivation process, iterative weighted least squares method can be applied, and the updated function is expressed as follows.

(15) $$\begin{array}{c} \begin{array}{c} \underset{C}{\arg\min}\theta \cdot \overset{G}{\underset{h=1}{\sum }}\Psi_{h}{C_{h}}^{2}\\ \text{subject to }B⊗C=A, \end{array} \end{array}$$

where *h* is the row number in the matrix, *G* is the number of columns of the point spread function, and Ψ is the weight obtained from the previous iteration. The equation can be optimized to Ψ_*h*_ = |*C*_*h*_^(*g* − 1)^|^−1^, and then, the optimized equation of *C* can be expressed as follows.

(16) $$\begin{array}{c} C^{\left(g\right)}=P_{g}B^{J}{\left({BP}_{g}B^{J}\right)}^{-1}A, \end{array}$$

where *P*_*g*_ is the diagonal matrix. In each iteration, only one iteration of weighted least squares is performed. When the point spread function *C* with high accuracy is estimated, the deconvolution method can be used to recover a clear ultrasound image from the blurred ultrasound image *A*. The recovery model can be expressed as follows.

(17) $$\begin{array}{c} \underset{B}{\arg\min}\overset{G}{\underset{q=1}{\sum }}\left(\frac{\lambda }{2}{\left(B⊗C-A\right)}_{q}^{2}+\overset{S}{\underset{s=1}{\sum }}{\left|B⊗U_{s}\right|}^{\alpha }\right), \end{array}$$

where *q* is the subscript of the pixel, *S* is the filter number, and *U* is the filter. ∑_*s*=1_^*S*^|*B* ⊗ *U*_*s*_|^*α*^ is used to express the gradient of *B* after convolution with the high-quality ultrasound image *B*. At this time, the semiquadratic splitting method is used to introduce auxiliary variables (here set to *V*_*q*_^1^*V*_*q*_^2^) to derive the model. The updated loss function can be expressed as follows.

(18) $$\begin{array}{c} \underset{Q,v}{\arg\min}\underset{q}{\sum }\left(\frac{J}{2}{\left(B⊗C-A\right)}_{q}^{2}+\frac{\eta }{2}\left({\left\|U_{q}^{1}B-V_{q}^{1}\right\|}_{2}^{2}+{\left\|U_{q}^{2}B-V_{q}^{2}\right\|}_{2}^{2}+{\left\|U_{q}^{1}B-V_{q}^{2}\right\|}_{2}^{2}\right)+{\left|V_{q}^{1}\right|}^{\alpha }+{\left|V_{q}^{2}\right|}^{\alpha }\right), \end{array}$$

where *η* is the weight value that is constantly changing in the regularization operation, expounding the difference between the auxiliary variable and the actual value. In the process of algorithm iteration, the weight will gradually change from low to high to achieve upgrading.

The article "Restoration Algorithm-Based Ultrasound Image in Evaluating the Effect of Dexmedetomidine on Patients with Neurological Disorder Anesthetized by Sevoflurane" was retracted in 2023. Reasons: signs of a paper mill; compromised peer review; unreliable results or conclusions.

### 2.6. Statistical Analysis

The SPSS 24.0 was used to process the data. Measurement data were expressed as the mean ± deviation (‾*x* ± *s*). Count data adopted the *χ*^2^ test. *P* < 0.05 was the threshold for significance.

## 3. Results

### 3.1. The General Data

As shown in Table 2, the differences in general data (age, gender, and weight) in the normal saline group, the control group, and the experimental group were not statistically significant (*P* > 0.05).

### 3.2. The Vital Signs in Different Time Periods during Anesthesia in the Three Groups of Patients

As shown in Figures 1–3, there was no statistically significant difference in the heart rate, mean arterial pressure, and blood oxygen saturation between the normal saline group, the control group, and the experimental group at different times during anesthesia (*P* > 0.05).

### 3.3. Operation Time, Extubation Time, and Recovery Time of the Three Groups of Patients

As shown in Figure 4, there was no statistically significant difference in the operation time between the three groups of patients (*P* > 0.05). The extubation time in the dexmedetomidine group was 10.6 ± 2.3 minutes, which was lower than the 12.1 ± 2.5 minutes of the saline group and 11.4 ± 2.1 minutes of the propofol group, and the difference was statistically significant (*P* < 0.05). The recovery time in the dexmedetomidine group was 8.4 ± 2.2 minutes, which was lower than 10.1 ± 2.3 minutes in the saline group and 9.0 ± 2.1 minutes in the propofol group, and the difference was statistically significant (*P* < 0.05).

The article "Restoration Algorithm-Based Ultrasound Image in Evaluating the Effect of Dexmedetomidine on Patients with Neurological Disorder Anesthetized by Sevoflurane" was retracted in 2023. Reasons: signs of a paper mill; compromised peer review; unreliable results or conclusions.

### 3.4. The Pain Scores and Agitation Scores of the Three Groups of Patients

As shown in Figure 5, the average pain score of patients in the dexmedetomidine group during the recovery period was 2.6 ± 0.7 points, which was lower than the 3.9 ± 0.6 points of the normal saline group and the 3.4 ± 0.8 points of the propofol group, and the difference was statistically significant (*P* < 0.05). The average agitation score in the dexmedetomidine group was 7.2 ± 2.4 points, which was lower than the 10.6 ± 3.7 points of the normal saline group and the 8.5 ± 2.3 points of the propofol group, and the difference was statistically significant (*P* < 0.05).

### 3.5. The Number of Cases of Vertigo in the Three Groups of Patients

As shown in Figure 6, a total of 13 patients in the dexmedetomidine group had vertigo during their recovery period, including 8 cases of central vertigo and 5 cases of peripheral vertigo, which were lower than the 15 cases and 11 cases in the normal saline group and 12 cases and 9 cases in the propofol group, and the difference was statistically significant (*P* < 0.05).

### 3.6. The Number of Cases of Nausea and Vomiting in the Three Groups of Patients

As shown in Figure 7, a total of 1 case of patients in the dexmedetomidine group had nausea and vomiting during the recovery period, accounting for 3%, which was lower than the 6 cases (20%) in the normal saline group and 4 cases (13%) in the propofol group, and the difference was statistically significant (*P* < 0.05).

### 3.7. The Hemodynamics of the Three Groups of Patients during the Recovery Period

As shown in Figure 8, the vascular ultrasound examination showed that the PSV of the left vertebral artery in the dexmedetomidine group during the recovery period was 67.7 ± 14.3 cm/s and that of the right was 67.9 ± 15.2 cm/s, which was lower than 81.5 ± 13.6 and 80.7 ± 11.6 cm/s in the normal saline group and 72.5 ± 12.9 and 73.4 ± 11.8 cm/s in the propofol group, and the difference was statistically significant (*P* < 0.05).

As shown in Figure 9, the vascular ultrasound examination showed that the EDV of the left vertebral artery in the dexmedetomidine group was 27.8 ± 6.7 cm/s during the recovery period and that of the right was 24.69 ± 5.9 cm/s, which was lower than 29.3 ± 6.8 and 28.9 ± 6.7 cm/s in the saline group and 28.6 ± 5.4 and 26.5 ± 5.1 cm/s in the propofol group, and the difference was statistically significant (*P* < 0.05).

As shown in Figure 10, the vascular ultrasound examination showed that the PSV of the left internal carotid artery in the dexmedetomidine group during the recovery period was 67.2 ± 13.9 cm/s and that of the right was 67.8 ± 12.7 cm/s, which was lower than the 74.3 ± 10.2 and 73.9 ± 12.5 cm/s in the normal saline group and 72.1 ± 11.4 and 73.5 ± 10.6 cm/s in the propofol group, and the difference was statistically significant (*P* < 0.05).

The article "Restoration Algorithm-Based Ultrasound Image in Evaluating the Effect of Dexmedetomidine on Patients with Neurological Disorder Anesthetized by Sevoflurane" was retracted in 2023. Reasons: signs of a paper mill; compromised peer review; unreliable results or conclusions.

As shown in Figure 11, the vascular ultrasound examination showed that the EDV of the left internal carotid artery in the dexmedetomidine group was 27.7 ± 5.3 cm/s during the recovery period and that of the right was 26.9 ± 4.9 cm/s, which was lower than 29.1 ± 4.3 and 29 ± 4.5 cm/s in the saline group and 28.8 ± 5.6 and 27.3 ± 4.7 cm/s in the propofol group, and the difference was statistically significant (*P* < 0.05).

As shown in Figure 12, vascular ultrasound examination showed that the RI of the left vertebral artery in the dexmedetomidine group during the recovery period was 0.6 ± 0.02 and that of the right was 0.71 ± 0.08, which was lower than the 0.84 ± 0.06 and 0.83 ± 0.05 in the saline group and 0.78 ± 0.07 and 0.82 ± 0.06 in the propofol group, and the difference was statistically significant (*P* < 0.05).

As shown in Figure 13, the vascular ultrasound examination showed that the RI of the left internal carotid artery in the dexmedetomidine group during the recovery period was 0.57 ± 0.04 and that of the right side was 0.58 ± 0.06, which was lower than 0.8 ± 0.04 and 0.81 ± 0.05 in the normal saline group and 0.76 ± 0.03 and 0.78 ± 0.05 in the propofol group, and the differences were statistically significant (*P* < 0.05).

### 3.8. Ultrasound Images before and after Applying the Restoration Algorithm

Figure 14 was the ultrasound images of a male patient, aged 35 years old, with symptoms of vertigo and nausea and vomiting after tonsillectomy. During the routine neck ultrasound examination, due to the aging of imaging equipment and other reasons, the ultrasound image was not clear and there was extra interference noise, which brought certain difficulties in the diagnosis and judgment of the disease. After the restoration algorithm was applied, the image obtained was clear and no unnecessary noise was noted.

## 4. Discussion

Sevoflurane is a kind of inhaled anesthetic that is widely used clinically. It is characterized by low aroma irritation, little effect on heart rate and hemodynamics, rapid anesthesia induction, and outstanding sedation and muscle relaxation effects [12, 13]. However, it can lead to neurological disorder in the postoperative recovery period, such as vertigo, headache, agitation, nausea and vomiting, and uneven hemodynamic indicators, affecting the physical and mental health of the patient [14, 15]. Therefore, it is necessary to use drugs during surgery to prevent adverse reactions caused by sevoflurane anesthesia. Dexmedetomidine acts on t12A receptors in the locus coeruleus area of the brainstem. It is a high-affinity *α*2 adrenergic receptor agonist, which can control the reflex of the autonomic nerves and has no effect on respiration and hemodynamic indicators. In addition, it has good sedative and analgesic effects [16, 17]. Hence, it is an ideal drug to reduce neurological disorder in patients under sevoflurane anesthesia during the recovery period.

The article "Restoration Algorithm-Based Ultrasound Image in Evaluating the Effect of Dexmedetomidine on Patients with Neurological Disorder Anesthetized by Sevoflurane" was retracted in 2023. Reasons: signs of a paper mill; compromised peer review; unreliable results or conclusions.

For neurological disorder-related symptoms, medical imaging is an important clinical examination method, among which ultrasound technology is the first choice. However, due to factors such as aging of imaging equipment, ultrasound images often have problems such as low resolution and redundant noise, which makes it impossible to accurately read image information [18]. In the study, the restoration algorithm was incorporated into the ultrasound imaging technology to improve the accuracy of imaging. 90 patients undergoing tonsillectomy were selected as research subjects and randomly divided into the normal saline group, propofol group, and dexmedetomidine group. The vascular ultrasound images for the neck were collected. The results showed that both propofol and dexmedetomidine had good sedation effect and good surgical effect when combined with sevoflurane inhalation for general anesthesia, consistent with the research results of Barends et al. [19], indicating that both propofol and dexmedetomidine are safe clinical anesthesia drugs. Besides, the dexmedetomidine group was superior to the normal saline group and the propofol group in extubation time, recovery time, average pain and agitation scores, and the number of cases of vertigo, nausea and vomiting, and hemodynamic indicators (PSV, EDV, and RI of bilateral vertebral arteries and internal carotid arteries), and the differences were statistically significant (*P* < 0.05). This indicates that during the period of recovery, the occurrence of the agitation is inevitable after using the two drugs, which was reflected in both groups of patients. However, the agitation score of the dexmedetomidine group was lower than that of the propofol control group. The reason may be that dexmedetomidine can inhibit sympathetic nerve activity, reduce serum concentration of adrenaline and norepinephrine, and keep hemodynamics stable. When the *α*2 adrenergic agonist binds to the *α*2 receptors in the spinal cord, it exerts its analgesic and calming effects, stopping the transmission of pain signals. As a result, the painful stimulus is reduced and the agitation response decreases. The experimental results were consistent with the conclusions of Sottas and Anderson [20] that dexmedetomidine had good sedative and analgesic effects. The ultrasound image processed by the restoration algorithm confirmed that dexmedetomidine can prevent neurological disorder caused by sevoflurane anesthesia, providing a reliable basis for the clinical treatment of pediatric anesthesia.

The article "Restoration Algorithm-Based Ultrasound Image in Evaluating the Effect of Dexmedetomidine on Patients with Neurological Disorder Anesthetized by Sevoflurane" was retracted in 2023. Reasons: signs of a paper mill; compromised peer review; unreliable results or conclusions.

## 5. Conclusion

In this experiment, an optimized restoration algorithm was incorporated into the ultrasound imaging system, to process the ultrasound images of patients anesthetized by sevoflurane for tonsillectomy. The results showed that children in the dexmedetomidine group were superior to the normal saline group and the propofol group in extubation time, recovery time, average pain and agitation scores, and the number of cases of vertigo, nausea and vomiting, and hemodynamic indicators (PSV, EDV, and RI of bilateral vertebral arteries and internal carotid arteries), and the differences were statistically significant, indicating that dexmedetomidine demonstrates good efficacy in preventing neurological disorder caused by sevoflurane anesthesia. However, some limitations should be noted. The sample size is small, which will reduce the power of the study. The follow-up requires large-scale multicenter randomized controlled trials to strengthen the findings of the study. Moreover, the application of restoration algorithm in ultrasonic imaging is not widespread enough and lacks deeper research. It is believed that with the development of science and technology, it will play a greater role in the field of medicine.

## Figures and Tables

**Figure 1:** Comparison of heart rate at different time periods during anesthesia in the three groups of patients. T1: before induction of anesthesia; T2: before intravenous administration; T3: 10 minutes after administration; T4: 30 minutes after administration; T5: after the operation.

**Figure 2:** Comparison of mean arterial pressure at different time periods during anesthesia in the three groups of patients. T1: before induction of anesthesia; T2: before intravenous administration; T3: 10 minutes after administration; T4: 30 minutes after administration; T5: after the operation.

**Figure 3:** Comparison of blood oxygen saturation at different time periods during anesthesia in the three groups of patients. T1: before induction of anesthesia; T2: before intravenous administration; T3: 10 minutes after administration; T4: 30 minutes after administration; T5: after the operation.

**Figure 4:** Comparison of operation time, extubation time, and recovery time of the three groups of patients. ∗ represented a statistically significant difference in the extubation time and recovery time of patients versus the dexmedetomidine group (*P* < 0.05).

The article "Restoration Algorithm-Based Ultrasound Image in Evaluating the Effect of Dexmedetomidine on Patients with Neurological Disorder Anesthetized by Sevoflurane" was retracted in 2023. Reasons: signs of a paper mill; compromised peer review; unreliable results or conclusions.

**Figure 5:** Comparison of pain scores and agitation scores of the three groups of patients. ∗ represented that the pain score and agitation score in the dexmedetomidine group were significantly different from those in the saline group and the propofol group (*P* < 0.05).

**Figure 6:** Comparison of the number of cases of vertigo in the three groups of patients. ∗ represented that the dexmedetomidine group was statistically different from the normal saline group and the propofol group in the number of cases of central vertigo and peripheral vertigo (*P* < 0.05).

**Figure 7:** Comparison of the number of cases of nausea and vomiting in the three groups of patients: the saline group, the propofol group, and the dexmedetomidine group. ∗ represented that the dexmedetomidine group was significantly different from the saline group and propofol group in the number of cases of nausea and vomiting (*P* < 0.05).

**Figure 8:** Comparison of PSV of bilateral vertebral arteries in the three groups of patients: the saline group (A), the propofol group (B), and the dexmedetomidine group (C). ∗ represented that the dexmedetomidine group was significantly different from that of the saline group and the propofol group in the PSV of bilateral vertebral arteries (*P* < 0.05).

**Figure 9:** Comparison of EDV of bilateral vertebral arteries in the three groups of patients: the saline group (A), the propofol group (B), and the dexmedetomidine group (C). ∗ represented that the dexmedetomidine group was significantly different from the saline group and the propofol group in the EDV of bilateral vertebral arteries (*P* < 0.05).

**Figure 10:** Comparison of PSV of bilateral internal carotid arteries in three groups of patients. ∗ represented that the dexmedetomidine group was significantly different from the saline group and the propofol group in the PSV of the bilateral internal carotid arteries (*P* < 0.05).

**Figure 11:** Comparison of EDV of bilateral internal carotid arteries in the three groups of patients. ∗ represented that the dexmedetomidine group was significantly different from the saline group and the propofol group in the EDV of the bilateral internal carotid arteries (*P* < 0.05).

**Figure 12:** Comparison of RI of bilateral vertebral arteries in the three groups of patients: the saline group (A), the propofol group (B), and the dexmedetomidine group (C). ∗ represented that the dexmedetomidine group was significantly different from the saline group and the propofol group in the RI of bilateral vertebral arteries (*P* < 0.05).

**Figure 13:** Comparison of RI of bilateral internal carotid arteries in the three groups of patients: the saline group (A), the propofol group (B), and the dexmedetomidine group (C). ∗ represented that the dexmedetomidine group was significantly different from the saline group and the propofol group in RI of bilateral internal carotid arteries (*P* < 0.05).

The article "Restoration Algorithm-Based Ultrasound Image in Evaluating the Effect of Dexmedetomidine on Patients with Neurological Disorder Anesthetized by Sevoflurane" was retracted in 2023. Reasons: signs of a paper mill; compromised peer review; unreliable results or conclusions.

**Figure 14:** Ultrasound images of the neck. (a) The original image. (b) The restored image.

**Table 1:** The scoring criteria for agitation.

Evaluation items	Score				
Can be awakened by gently shaking	None (4 points)	Poor (3 points)	Good (2 points)	Very good (1 point)	Excellent (0 points)
Obey instructions	None (4 points)	Poor (3 points)	Good (2 points)	Very good (1 point)	Excellent (0 points)
Emotional upset	None (0 points)	Light (1 point)	Medium (2 points)	Severe (3 points)	Extremely severe (4 points)
Need to be tied up	None (0 points)	Light (1 point)	Medium (2 points)	Severe (3 points)	Extremely severe (4 points)
Try to attack the paramedics	None (0 points)	Light (1 point)	Medium (2 points)	Severe (3 points)	Extremely severe (4 points)

**Table 2:** Comparison of general data of the three groups of patients.

Basic clinical information	Normal saline group	Propofol group	Dexmedetomidine group
Age (year)	43.8 ± 11.5	43.3 ± 11.7	44.5 ± 11.2
Gender (male/female)	18/12	16/14	15/15
Weight (kg)	64.8 ± 12.3	65.7 ± 12.6	63.9 ± 11.7

## Data Availability

The data used to support the findings of this study are available from the corresponding author upon request.

## References

[1] Konishi Y., Evered L. A., Scott D. A., Silbert B. S. (2018). Postoperative cognitive dysfunction after sevoflurane or propofol general anaesthesia in combination with spinal anaesthesia for hip arthroplasty. *Anaesthesia and Intensive Care*.

[2] van der Griend B. F., Vincent A. R., Kennedy R. R. (2019). Observational audit of sevoflurane consumption during paediatric anaesthesia. *Anaesthesia and Intensive Care*.

[3] Tan D., Xia H., Sun S., Wang F. (2019). Effect of ancillary drugs on sevoflurane related emergence agitation in children undergoing ophthalmic surgery: a Bayesian network meta-analysis. *BMC Anesthesiology*.

[4] Amorim M. A., Govêia C. S., Magalhães E., Ladeira L. C. A., Moreira L. G., Miranda D. B. (2017). Effect of dexmedetomidine in children undergoing general anesthesia with sevoflurane: a meta-analysis. *Brazilian Journal of Anesthesiology*.

[5] Ebrahimi A., Eslami J., Darvishi I., Momeni K., Akbarzadeh M. (2020). Investigation of the role of complementary medicine on anxiety of patients before and after surgery: a review study. *Nursing Practice*.

[6] Tang C. L., Li J., Zhang Z. T. (2018). Neuroprotective effect of bispectral index-guided fast-track anesthesia using sevoflurane combined with dexmedetomidine for intracranial aneurysm embolization. *Neural Regeneration Research*.

The article "Restoration Algorithm-Based Ultrasound Image in Evaluating the Effect of Dexmedetomidine on Patients with Neurological Disorder Anesthetized by Sevoflurane" was retracted in 2023. Reasons: signs of a paper mill; compromised peer review; unreliable results or conclusions.

[7] Han M., Kang F., Yang C. (2020). Comparison of adrenaline and dexmedetomidine in improving the cutaneous analgesia of mexiletine in response to skin pinpricks in rats. *Pharmacology*.

[8] Yang Z., Song G., Hu W., Dang X., Haijuan G., Yu J. (2018). Pharmacological analysis of dexmedetomidine hydrochloride in pediatric anesthesia during magnetic resonance imaging. *Pakistan Journal of Pharmaceutical Sciences*.

[9] Lv Z. H., Yang H., Singh A. K., Manogaran G., Lv H. (2021). Trustworthiness in industrial IoT systems based on artificial intelligence. *IEEE Transactions on Industrial Informatics.*.

[10] Xie S. X., Yu Z. C., Lv Z. H. (2021). Multi-disease prediction based on deep learning: a survey. *Computer Modeling in Engineering & Sciences*.

[11] Wan Z., Dong Y., Yu Z., Lv H., Lv Z. (2021). Semi-supervised support vector machine for digital twins based brain image fusion. *Frontiers in Neuroscience*.

[12] Kennedy R. R., Hendrickx J. F., Feldman J. M. (2019). There are no dragons: low-flow anaesthesia with sevoflurane is safe. *Anaesthesia and Intensive Care*.

[13] Varnäs K., Finnema S. J., Johnström P. (2021). Effects of sevoflurane anaesthesia on radioligand binding to monoamine oxidase-B in vivo. *British Journal of Anaesthesia*.

[14] Wu X., Cao J., Shan C. (2019). Efficacy and safety of propofol in preventing emergence agitation after sevoflurane anesthesia for children. *Experimental and Therapeutic Medicine*.

[15] Benarroch E. E. (2020). Physiology and pathophysiology of the autonomic nervous system. *CONTINUUM: Lifelong Learning in Neurology*.

[16] Chikuda M., Sato K. (2019). Effects of dexmedetomidine on porcine pulmonary artery vascular smooth muscle. *BMC Anesthesiology*.

[17] Zhang T., Yu Y., Zhang W., Zhu J. (2019). Comparison of dexmedetomidine and sufentanil as adjuvants to local anesthetic for epidural labor analgesia: a randomized controlled trial. *Drug Design, Development and Therapy*.

[18] Bevan R. L. T., Zhang J., Budyn N., Croxford A. J., Wilcox P. D. (2019). Experimental quantification of noise in linear ultrasonic imaging. *IEEE Transactions on Ultrasonics, Ferroelectrics, and Frequency Control*.

[19] Barends C. R., Absalom A., van Minnen B., Vissink A., Visser A. (2017). Dexmedetomidine versus midazolam in procedural sedation. A systematic review of efficacy and safety. *PLoS One*.

[20] Sottas C. E., Anderson B. J. (2017). Dexmedetomidine: the new all-in-one drug in paediatric anaesthesia?. *Current Opinion in Anaesthesiology*.

